The article "The Close Relationship between Large Bowel and Heart: When a Colonic Perforation Mimics an Acute Myocardial Infarction" was published in 2018. Journal: Case Rep Surg.

# The Close Relationship between Large Bowel and Heart: When a Colonic Perforation Mimics an Acute Myocardial Infarction

**DOI:** 10.1155/2018/8020197

**Published:** 2018-07-16

**Authors:** Maria Francesca Secchi, Carlo Torre, Giovanni Dui, Francesco Virdis, Mauro Podda

**Affiliations:** ^1^Department of Emergency and Acute Care Medicine, San Francesco Hospital, Nuoro, Italy; ^2^Department of Gastrointestinal Endoscopy, San Francesco Hospital, Nuoro, Italy; ^3^Department of Radiology, San Francesco Hospital, Nuoro, Italy; ^4^Department of Trauma and Emergency Surgery, King's College Hospital, London, UK; ^5^Department of General, Emergency, and Robotic Surgery, San Francesco Hospital, Nuoro, Italy

## Abstract

Colonoscopic perforation is a serious and potentially life-threatening complication of colonoscopy. Its incidence varies in frequency from 0.016% to 0.21% for diagnostic procedures, but may be seen in up to 5% of therapeutic colonoscopies. In case of extraperitoneal perforation, atypical signs and symptoms may develop. The aim of this report is to raise the awareness on the likelihood of rare clinical features of colonoscopic perforation. A 72-year-old male patient with a past medical history of myocardial infarction presented to the emergency department four hours after a screening colonoscopy with polypectomy, complaining of neck pain, retrosternal oppressive chest pain, dyspnea, and rhinolalia. Right chest wall and cervical subcutaneous emphysema, pneumomediastinum, pneumoretroperitoneum, and bilateral subdiaphragmatic free air were reported on the chest and abdominal X-rays. The patient was treated conservatively, with absolute bowel rest, total parental nutrition, and broad-spectrum intravenous antibiotics. Awareness of the potentially unusual clinical manifestations of retroperitoneal perforation following colonoscopy is crucial for the correct diagnosis and prompt management of colonoscopic perforation. Conservative treatment may be appropriate in patients with a properly prepared bowel, hemodynamic stability, and no evidence of peritonitis. Surgical treatment should be considered when abdominal or chest pain worsens, and when a systemic inflammatory response arises during the conservative treatment period.

## 1. Introduction

Colonoscopy has become a standard tool for colorectal cancer screening worldwide. As endoscopists have gained increased experience performing the procedure, the incidence of colonoscopic complications shows a decreasing trend [1]. Overall morbidity following colonoscopy is 0.2% and 1.2% for diagnostic and therapeutic procedures, respectively [2].

In particular, colonoscopic perforation (CP) is one of the most serious and potentially life-threatening complications of colonoscopy.

CP is usually categorized into intraperitoneal, extraperitoneal, or intra- and extraperitoneal. Extraperitoneal CP is extremely rare. This occurs when the perforation site is located in the segments of the colonic wall which are attached to the extraperitoneal planes, such as the posterior walls of the ascending, descending sigmoid, rectosigmoid colon, and rectum [3].

In case of extraperitoneal perforation, atypical signs and symptoms, such as rhinolalia, pneumomediastinum, pneumoretroperitoneum, subcutaneous emphysema, dyspnea, and chest discomfort may develop [4, 5].

We present the clinical case of a patient admitted to the emergency department (ED) for cardiac-type chest pain, abdominal and thoracic subcutaneous emphysema, and rhinolalia, following operative colonoscopy and resection of a polypoid neoplasm of the cecum. The aim of this report is to raise the awareness on the likelihood of these rare clinical features of CP.

## 2. Case Presentation

A 72-year-old male patient presented to the emergency department (ED) complaining of neck pain, retrosternal oppressive chest pain, and progressive dyspnea, reporting also a change of the voice with rhinolalia. The patient's past medical history was significant for coronary heart disease. The patient was diagnosed with ST-elevation myocardial infarction (STEMI) in 2001, and non-ST-elevation myocardial infarction (NSTEMI) in 2006. A permanent pacemaker was positioned in 2009 for sinus node dysfunction.

In order to investigate iron deficiency anemia and a positive immunochemical fecal occult blood, the patient had undergone an outpatient screening colonoscopy four hours earlier.

The colonoscopy revealed three potential neoplastic lesions. The first one was a sessile polyp of 10 mm in diameter sited in the cecum, close to the ileocecal valve. It was removed with the diathermic loop, after infiltration of the mucosa with adrenaline.

A further two polyps were found in the ascending colon, both of about 7 mm in diameter.

As the cecal polyp exeresis was complicated by bleeding, a hemostatic clip was placed near the ileocecal valve. No obvious perforations were seen during the procedure (Figure 1), and no symptoms related to perforations, such as abdominal distension, abdominal and chest pain, or dyspnea were identified at the physical examination immediately after the procedure.

However, two hours after the completion of the procedure, the patient started complaining of abdominal, chest, and neck pain and shortness of breath.

Additional information was obtained from the endoscopist who performed the procedure. He mentioned extensive diverticular disease of the sigmoid colon and good mechanical preparation (Boston Bowel Preparation Scale: BBPS 2-3-3).

On ED arrival, the patient was apyretic. He had a blood pressure of 140/80 mmHg, a heart rate of 65 bpm, and an oxygen saturation on room air of 96%. The patient described the chest pain as a constriction, not radiated, and exacerbated by deep breaths.

The airway was intact and he was able to talk, although with rhinolalia. The abdomen was slightly distended and soft, although abdominal pain without signs of peritoneal irritation was located mainly on the right quadrants.

Subcutaneous emphysema, with a clear crepitus on palpation, was apparent on the neck, right anterior chest wall, and anterior and right lateral abdominal wall.

Due to the reported anamnesis of cardiovascular pathology, an electrocardiogram was performed. It showed a T wave inversion in the inferior and lateral leads, without any pacemaker activity (Figure 2). However, cardiac enzymes, as well as blood tests, inflammatory markers, and hemogas analysis were all unremarkable. Neck, chest, and abdominal X-rays were then requested to rule out the clinical suspicion of CP.

Right chest wall and cervical subcutaneous emphysema, pneumomediastinum, pneumoretroperitoneum, and bilateral subdiaphragmatic free air were reported on the chest and abdominal X-rays (Figure 3).

The abdominal and lower thorax contrast-enhanced computed tomography (CT) scan revealed pneumoperitoneum and pneumoretroperitoneum, mainly located at the epimesogastrium, at the right anterior and posterior pararenal and perihepatic spaces, as well as diverticulosis of the sigmoid colon (Figure 4). No questionable findings, such as an obvious intestinal perforation, peritoneal fluid, or radiological signs of peritonitis, were noted.

In view of the clinical and radiological findings, the patient's good general condition and hemodynamic stability, and the absence of peritoneal irritation and signs of inflammatory syndrome, the patient was admitted to the surgical department and treated conservatively, with absolute bowel rest, total parental nutrition, broad-spectrum intravenous antibiotics (ciprofloxacin 500 mg × 2 and metronidazole 500 mg × 3), and symptomatic care.

Vital signs on the day after the procedure included a blood pressure of 125/80 mmHg, a pulse rate of 75 bpm, a respiratory rate of 16 breaths/min, and a body temperature of 36.7°C. Follow-up chest and abdominal X-rays exhibited a resolving pneumomediastinum and pneumoretroperitoneum 48 hours after the admission. C-reactive protein was slightly raised to 0.86 mg/dl, without any other laboratory sign of inflammation. The patient's subcutaneous emphysema markedly resolved on the third postprocedure day.

Diet was started from water intake at the 5th day after the procedure, and oral antibiotics were administered instead of intravenous antibiotics. The patient recovered uneventfully and was discharged on the 12th day after admission.

The condition of the patient was observed in the outpatient clinic one week after his leaving the hospital, and was confirmed to be fully recovered without any further complications.

## 3. Discussion

### 3.1. Epidemiology and Pathogenesis

The incidence of CP varies in frequency from 0.016% to 0.21% for diagnostic procedures, but may be seen in up to 5% of therapeutic colonoscopies [6, 7].

Many factors, related both to the patient (advanced age, diabetes, chronic pulmonary disease, myocardial infarction, cerebrovascular disease, congestive heart failure, renal insufficiency, peripheral vascular disease, diverticular disease, and previous abdominal surgery) and to the procedure itself (therapeutic colonoscopy with polypectomy, pneumatic dilatation, and endoscopic mucosal resection) may be related to the incidence of CP [8]. Convincing evidence shows that with polypectomies the risk of CP rises to 0.3–1%, and with hydrostatic balloon dilatation of colonic strictures, higher rates (4-5%) may be expected [9, 10].

CP may be caused by one of the following three mechanisms: (1) mechanical trauma by instrumentation, (2) barotrauma by excessive air inflation, and 3) thermal injury by electric current during colonoscopy [11].

The sigmoid colon is the most affected site of CP, followed in frequency by the rectum [12, 13].

Although the cecum and the ileocecal valve are rarely involved in perforations, the thin wall layer and the large lumen of the cecum make this colonic segment more vulnerable to injury by polypectomy, as reported in the present case [14].

Since the peritoneum, retroperitoneum, mediastinum, and thorax are anatomically connected, when perforation occurs, intraluminal compressed air may escape into either the peritoneum and the retroperitoneum. Once in the retroperitoneum, air may travel along the mesentery, large vessels, and through the diaphragmatic hiatus, and then further spread to the mediastinum and subcutaneous tissues [15]. Eventual rupture of the mediastinal pleura allows air to decompress into the pleural cavity and cause pneumothorax. Pneumothorax can also develop when the pneumoperitoneum extends to the intrapleural space through the diaphragmatic fenestrations [16].

In the present report, extraluminal air probably entered the body due to a cecal perforation following polypectomy, leading to an extremely rare combined pattern of intra- and extraperitoneal perforation.

### 3.2. Clinical Presentation

Key points from diagnosis to treatment of CP are summarized in Table 1.

The most common presenting symptom after CP is abdominal pain, although clinical manifestations may be variable according to the location, size, mechanism of the perforation, the extent of the soiling, and bowel preparation.

If the perforation site is in the retroperitoneum, peritoneal irritation signs may not be evident, resulting in unusual presentation, as in the current report. The review of the literature published by Cirt et al., found 24 reported cases of retroperitoneal CP with various clinical presentations. Among them, 14 cases were associated with polypectomies. Cases involving both intraperitoneal and extraperitoneal CP following colonoscopy were extremely rare, with only 11 such cases reported [10].

CP into the retroperitoneum can spread to the other areas, resulting in unusual clinical manifestations which offer important clues for early diagnosis. Voice changes, such as hoarseness and rhinolalia, have been reported as rare signs of CP, which may be caused by changes in the anatomy of the pharyngeal region due to the presence of emphysema [17, 18].

### 3.3. Diagnosis

To avoid any delay before the correct diagnosis, clinicians should suspect a CP if any patient recently submitted to colonoscopy develops subcutaneous emphysema, fever, and abdominal or chest pain. These clinical features should be kept in mind even if the patient presents the symptoms several days after the procedure [12, 13].

The recent review conducted by Tiwari et al. revealed that about 50% of CPs are detected immediately or within 1 hour, whereas 30% are found within 1–24 hours and 20% found after 24 hours from the procedure [16].

When CP is suspected, key diagnostics are chest and abdominal X-rays. These may demonstrate pneumoperitoneum, pneumomediastinum, pneumoretroperitoneum, pneumothorax, and subcutaneous emphysema.

However, in cases of retroperitoneal perforation, free air might not be visible on plain X-rays. In such cases, CT scan, eventually with double contrast (intravenous and rectal) is a more effective diagnostic modality for detecting pneumoretroperitoneum [19, 20].

CT is also mandatory in those patients with CP who are eligible for conservative management because it can detect not only a small amount of free intra-abdominal gas but also the presence of free fluid and other typical features of peritonitis [21].

### 3.4. Treatment Strategies

Historically, surgery with explorative laparotomy was the mainstay of treatment for the majority of patients. However, the likelihood of nonoperative treatment has increased. Conservative treatment should be reserved for patients in good general conditions, without any sign of generalized peritonitis, perforation unnoticed by the endoscopist, a good degree of bowel preparation, early detection of the CP, and no underlying disease requiring surgery [13, 21].

The conservative approach involves intravenous fluids, bowel rest, and intravenous administration of broad-spectrum antibiotics [10].

The overall success rate of a nonoperative treatment for CP ranges from 33% to 73%, and small perforations caused by therapeutic colonoscopy have been shown to have a better success rate with medical treatment [12].

Conversely, primary surgical management is recommended in patients with extensive peritoneal contamination, poor general condition, hemodynamic instability, and presence of concurrent colonic lesions which require surgery [22].

The type of surgical treatment should be tailored on a case-by-case basis. Simple closure with sutures may be appropriate in the case of small CP (<50% of bowel circumference), without significant fecal contamination and concomitant intestinal pathology requiring bowel resection [12].

Conversely, segmental bowel resection is required when the perforation is large, or when the primary closure of the perforation could compromise the lumen, or when there is concomitant colorectal pathology (cancer, severe colonic stricture, and large sessile polyp) that requires bowel resection. The choice between bowel resection with primary anastomosis and Hartmann's procedure is related to the grade of intra-abdominal contamination, the timing of the diagnosis, and the general condition of the patient [12].

All patients under nonoperative treatment should be closely monitored. If conservative management is successful, the patient's clinical appearance should improve gradually within the first 48 hours, as reported also in our case [12]. Conversely, when pain worsens, or a systemic inflammatory response manifests with fever, tachycardia, tachypnea, and elevated inflammatory markers, complicated intra-abdominal infections (intra-abdominal abscesses or generalized fecal peritonitis) should be suspected, and thus further investigations and prompt surgical treatment should be considered [13].

Endoscopic clipping followed by conservative treatment has been recently reported and could be a valid approach in patients with small lesions and without signs of peritonitis [11]. In general, the size of the perforation suitable for endoscopic closure is less than 10 mm, but some reports showed successful endoscopic repairs of perforations larger than 10 mm [12]. A review of 75 cases of CP repaired by endoclipping, by Trecca et al. in 2008, reported a success rate of 69%–93%. Early recognition of the CP, prompt complete endoscopic repair, and good bowel preparation are the keys to the success of endoscopic treatment for CP [23].

## 4. Conclusion

Awareness of the potentially unusual clinical manifestations of retroperitoneal perforation following colonoscopy is crucial for the correct diagnosis and prompt management of CP.

Treatment strategies for patients with CP should be patient-tailored, based on clinical presentation, patient's general condition, grade of colonic preparation, nature of perforation, and underlying colorectal pathologies.

Conservative treatment may be appropriate in patients with a properly prepared bowel, hemodynamic stability, and no evidence of peritonitis. However, prompt surgical treatment should be considered when abdominal or chest pain worsens, and when a systemic inflammatory response arises during the conservative treatment period.

## Figures and Tables

**Figure 1:** Colonoscopic finding. No definite perforation is seen. Hemostatic clipping and hot biopsy coagulation near the ileocecal valve were done.

**Figure 2:** Electrocardiogram showing T wave inversion in the inferior and lateral leads.

**Figure 3:** (a) Abdominal X-ray showing subcutaneous emphysema, pneumomediastinum, pneumoretroperitoneum, and right subdiaphragmatic free air (black arrow). (b) Chest X-ray showing pneumomediastinum (red arrow). (c) Neck X-ray showing right cervical subcutaneous emphysema (green arrow).

**Figure 4:** Abdominal CT scan showing pneumoperitoneum and pneumoretroperitoneum (a, b), mainly located at the epimesogastrium, at the right anterior and posterior pararenal and perihepatic spaces (c) (black arrows, red arrow).

**Table 1:** Key points for early diagnosis and treatment of patients with CP.

Clinical features	Diagnostic workup	Treatment strategies
(1) Abdominal pain (diffuse or localized) (2) Abdominal tenderness (diffuse or localized) (3) Abdominal guarding (diffuse or localized) (4) Ileus (5) Chest pain (6) Voice changes (hoarseness, rhinolalia) (7) Subcutaneous emphysema (abdomen, chest, and neck) (8) Fever (>38°C) (9) Tachycardia (>100 beats/min) (10) Tachypnea (>20 breaths/min) (11) Oliguria (urine output <21 ml/h)	(1) *Blood tests* (i) Leukocytosis (ii) Neutrophilia (2) *Inflammatory markers* (i) High levels of C-reactive protein (ii) High levels of procalcitonin (3) *Abdominal X-ray* (i) Pneumoperitoneum (ii) Pneumoretroperitoneum (iii) Subcutaneous emphysema (4) *Chest X-ray* (i) Pneumothorax (ii) Pneumomediastinum (iii) Subcutaneous emphysema (5) *Abdominal CT scan with oral and rectal contrast* (i) Typical features of peritonitis (ii) Free intra-abdominal gas (iii) Free intra-abdominal fluid (iv) Peritoneal and mesenteric thickening	(1) *Conservative treatment (intravenous fluids, bowel rest, and intravenous administration of broad-spectrum antibiotics)* (i) Patients in good general conditions (ii) No signs of generalized peritonitis (iii) Perforation unnoticed by the endoscopist (iv) Good degree of bowel preparation (v) Early detection of the CP (vi) No underlying disease requiring surgery (2) *Surgery (simple closure with sutures)* (i) Small CP < 50% of bowel circumference (ii) No fecal contamination (iii) No concomitant intestinal pathology requiring bowel resection (3) *Colonic resection (Hartmann's versus colectomy and primary anastomosis)* (i) Depending on the grade of intra-abdominal contamination and the general condition of the patient (4) *Endoscopic clipping followed by conservative treatment* (i) Early recognition of the CP (ii) Small CP < 10 mm (iii) No signs of peritonitis (iv) Good bowel preparation

## Abbreviations

CP: Colonic perforation
ED: Emergency department
STEMI: ST-elevation myocardial infarction
NSTEMI: Non-ST-elevation myocardial infarction
CT: Computed tomography.
